The article "Measuring the Effect of Vision on the Synergy of Lower Extremity Muscles during Walking using Nonnegative Matrix Factorization (NNMF) Algorithm Method" was published in 2023. Journal: Appl Bionics Biomech.

# Measuring the Effect of Vision on the Synergy of Lower Extremity Muscles during Walking using Nonnegative Matrix Factorization (NNMF) Algorithm Method

**DOI:** 10.1155/2023/5501871

**Published:** 2023-04-18

**Authors:** Nasim Safari, Mahboubeh Alemzadeh, Mahdi Majlesi, Nader Farahpour, Muharram Mansoorizadeh

**Affiliations:** ^1^Department of Kinesiology, Faculty of Sport Sciences, Bu-Ali Sina University, Hamedan, Iran; ^2^Department of Sport Biomechanics, Faculty of Humanities, Islamic Azad University, Hamedan Branch, Hamedan, Iran; ^3^Computer Engineering Department, Bu-Ali Sina University, Hamedan, Iran

## Abstract

**Introduction:**

Lack of visual information in blind people during walking can affect the choice of muscle synergy from among the many incoming messages that reach the central nervous system (CNS). This study aimed to determine the effect of vision on the synergy of lower limb muscles during walking using the nonnegative matrix factorization algorithm (NNMF).

**Methods:**

Ten blind people and 10 people with normal vision participated in this study. Activities of involved muscles were recorded during walking. Muscle synergy matrix and synergy activation coefficient were calculated using the NNMF algorithm, while the variance accounted for criterion was used to determine the number of synergies required during walking. In order to assess the similarity of muscle synergy pattern and the relative weight of each muscle in each synergy in each group, Pearson correlation and independent samples *t*-test at a significance level of *α* ≤ 0.05 were used.

**Results:**

Four muscle synergies were extracted from EMG data during walking. The first (*r* = 0.431) and the second (*r* = 0.457) synergy patterns showed a moderate correlation between the two groups. However, the third (*r* = 0.302) and the fourth (*r* = 0.329) synergy patterns showed a weak correlation between the two groups. In the blind group, the relative weight of the muscles in the first synergy was significant for the external extensor muscle (*P* = 0.023), and in the second synergy for the biceps femoris. Also, in the third synergy, the relative weight was found to be significant in none of the muscles. In the fourth synergy, however, the relative weight of external extensor muscle in the blind group showed a significant decrease, as compared to the group with normal vision.

**Conclusions:**

These changes can be the strategy of the CNS to preserve the optimal functioning in the motor system of blind people.

## 1. Introduction

Synergy theory is one of the most interesting hypotheses about motion control, which considers the central nervous system (CNS) as a model for controlling motor function. This model reduces the degree of CNS freedom in controlling muscle groups and movements and allows muscle groups to be activated as a whole. This model shows muscle groups as a module or synergy for movement control [1, 2]. The motion control system always organizes the body's activities in such a way that the highest efficiency is achieved with the least amount of muscle fatigue [3, 4]. Synergy creates a coordinated and optimal movement in terms of energy consumption by creating a coordinated relationship between a group of muscles involved in the desired activity. The main importance of this issue is the simplification of the body movement control system. Based on the synergy hypothesis, motor bases will be organized at the level of the spinal cord and will result in a reduction in muscle group contraction [5] so that the body control system can use a small number of synergies instead of hundreds of muscles to control movement. According to studies, researchers believe that muscles are not independently controlled by the brain but are controlled as a group of muscles and are placed in synergy groups by coefficients of activity. This is referred to as muscle synergy [6], and these synergies cause specific motor behaviors [7]. Humans use this unique neuromuscular-skeletal mechanism to achieve the desired result, which is to performing a specific movement with complete accuracy [8]. Walking is the result of a complex interaction between the brain, spinal cord, and peripheral nerves that require well coordinate leg joints and body muscles; since sensory inputs are the basis of human movement control, especially for walking. Due to the lack of visual information, blind people face numerous limitations in cognitive and motor functioning. Careful posture maintenance is one of the characteristics of gait in blind people, and changes therein can reflect the strategies that blind people adopt to maintain posture stability [9]. Congenitally blind people have never received visual stimuli; however, despite the lack of vision from the beginning, they have learned motor activity and motor skills such as orientation and motor activities in daily life, although their movement patterns may be different from normal people. Therefore, by accumulating information about gait patterns and the effect of vision in individuals, it is possible to identify the problems they face during walking [10]. In addition, the effect of internal visual acuity on people during walking can be examined. Given that sensory inputs, including visual inputs, provide the information required for controlling movement, especially walking [11], and that in each synergy, different patterns of muscle activities also depend on sensory and motor inputs. It has also been shown that walking follows synergistic control [12, 13]. Therefore, impairment of sensory inputs can be one of the main causes of changes in the selection of muscle synergy in the CNS. In a study by Yoshida et al. [14], the effect of vestibular disorders on changes in synergy pattern when walking was investigated, and it was shown that muscle synergy patterns would not change significantly. In several studies, four muscle synergies have been reported during human walking in different conditions, including speed of walking [12, 15] and walking with different loads [16], where no change in the number of synergy patterns has been observed as compared to those in the normal gait. In their study, Martino et al. [17] showed that the number of muscle synergies in sitting-to-standing movement did not differ between people with closed eyes and open eyes. They identified four synergies for both groups. This suggested that the nervous system is able to adopt a different motor strategy for the long-term adaptation of muscle activities under unstable conditions [17]. In other words, humans may depend on other sensory inputs when they suffer from vestibular and vision disorders. Despite the studies conducted in the field of synergies during walking, the analysis of synergy in blind people has not been investigated. Since muscle synergy can inspire the design of systems for rehabilitation that are as similar as possible to the natural pattern of the body. The aim of this study was to extract the muscle synergy in the muscles of the lower extremities and during walking in the blind and normal vision individuals and to determine the number of muscle synergies and the relative weight of muscle activities involved in gait using the nonnegative matrix decomposition. Lack of visual input in blind people, which leads to the adoption of specific posture strategies, can also affect the number of muscle synergies, the relative weight of muscle activity, and muscle function during walking; It is not known how muscle synergies change in condition of lack of visual information during walking?

The article "Measuring the Effect of Vision on the Synergy of Lower Extremity Muscles during Walking using Nonnegative Matrix Factorization (NNMF) Algorithm Method" was published in 2023. Journal: Appl Bionics Biomech.

## 2. Method

### 2.1. Participants

The statistical population of this study included blind people and people with normal vision living in Hamedan. Using G^*∗*^ Power software with *α* = 0.05 and statistical power of 80% (35, 34), it was decided that at least 20 subjects were required for this study, of which 10 were blind men as a blind group and 10 men with normal vision as the group with normal vision. The people participated in this study voluntarily.

As shown in Table 1, people with normal vision were not significantly different from blind people in terms of demographic characteristics. The blind group in this study was blind from birth, and also none of the participants in both groups had no history of continuous exercise in the past 2 years. Individuals with lower extremity injuries or neurological and orthopedic diseases during the past 6 months were excluded from the study. The subjects completed the consent form to participate in the test, and then the procedure was fully explained to the subjects. The protocol of the study was approved by the Ethics Committee of Hamedan University of Medical Sciences, Hamedan, Iran (p/16/35/9/5827).

### 2.2. Apparatus and Protocol

In order to measure the electrical activity of muscles, a 16-channel electromyography device model BTS Free EMG 300, BTS, Italy, with disposable bipolar electrodes (with a diameter of 12 mm, the center-to-center distance of 20 mm) was used. Electromyography signals with a frequency of 1,000 Hz, CMRR > 110 ds, and gain equal to 1,000 were recorded. To install the electrodes, all the recommendations of the International Electromyography Association were followed [18]. For this purpose, first, the excess hair at the electrode installation spot was shaved and then cleaned with a cotton swab dipped in 5% isopropyl alcohol. The position of the electrodes was parallel to the direction of the muscle fibers. Electrodes were placed on the skin in the gastrocnemius medialis (GA), tibialis anterior, vastus lateral (VL), gluteus maximus, and biceps femoris (BF) muscles on the side of the body. These muscles are the main contributors to human walking [19]. Subjects from both groups were asked to walk the designated 12 m route at their normal pace. All subjects underwent soft movements for about 5 min before the start of the test and walked the desired path several times. Blind people also went through the path several times using their white canes to get acquainted with the path. During the main test, blind people were assured that they would be given verbal warnings if they deviated from the course or in the event of any collision with objects. Thus blind people did not have to worry about hitting objects or falling. In each of the variables, the average score obtained from three repetitions was considered for statistical analyses.

### 2.3. Data Analysis

EMG Graphing software was used to analyze the electromyography data. To perform linear envelope, first, a filter with a frequency of 10–500 was used, and then the signals were full wave rectified and refined again with a 6 Hz Butterworth filter [20]. The submaximal method was used to normalize the data. First, the maximum activity of the muscles in each cycle was calculated, and then each data point was divided into the maximum activity of the muscles in each cycle to obtain muscle activity based on a percentage of the maximum activity of the muscles per cycle [21]. At the end, it was time-normalized through cubic interpolation and divided into 101 points. All analyses were carried out through MATLAB. In order to calculate muscle synergy, data for each individual in the two groups were stored in the 101 × 5 matrix. Negative matrix analysis or NNMF was used to extract synergies from electromyogram signals of a nonnegative nature. Negative factorization of the matrix is an algorithm for decomposing the information matrix into two negative matrices with lower dimensions and a method for quantifying the concept of synergy using Equation (1) [22].

(1) $$\begin{array}{c} M=HW. \end{array}$$

Using this model, the electromyography signal matrix *M* (number of frames × number of muscles) is divided into two matrices, *H* (number of frames × number of synergies), which shows the synergy activation coefficients, and *W* (number of synergies × number of muscles), which shows the muscle synergy matrix.

The article "Measuring the Effect of Vision on the Synergy of Lower Extremity Muscles during Walking using Nonnegative Matrix Factorization (NNMF) Algorithm Method" was published in 2023. Journal: Appl Bionics Biomech.

### 2.4. Calculating Variance Accounted For (VAF)

VAF is calculated by Equation (2), where EMG_*t*_^rec^ is the reconstructed electromyography signal, and EMG_*t*_^exp^ is the input or main electromyography signal in the *t*-frame [23].

(2) $$\begin{array}{c} VAF=1-\frac{\sum_{t=1}^{101}{EMG}_{t}^{rec}-{EMG}_{t}^{exp}}{\sum_{t=1}^{101}{EMG}_{t}^{exp}}. \end{array}$$

The analysis for each subject began by assuming that only one synergy was needed for electromyography reconstruction. If VAF was >0.9 for each of the five muscles, it was concluded that additional synergies were not needed [23].

### 2.5. Statistical Analysis

Shapiro–Wilk test was used to test the normality of the data and the possibility of using parametric tests. Pearson correlation was used to evaluate the similarity of the muscle synergy pattern in the two groups. If the degree of correlation in each synergy is close to one, it indicates the similarity of the pattern of muscle synergies (0.0–0.29: small similarity, 0.3–0.69: moderate similarity, 0.7–1: high similarity) [24]. Relative muscle weight in both groups and VAF data were analyzed using independent samples *t*-test. All stages of statistical analysis of data were performed using SPSS software version 21 with a significance level of *α* < 0.05.

## 3. Results

### 3.1. VAF Values for Muscles in the Two Groups

VAF criterion was used to determine the number of synergies based on the number of muscles in the NMF algorithm. As shown in Table 2, VAF values for two groups showed that four synergies were suitable for the reconstruction of the main signal and all of VAF had a value >0.9. There was also no significant statistical difference in the values of VAF for both groups.

The article "Measuring the Effect of Vision on the Synergy of Lower Extremity Muscles during Walking using Nonnegative Matrix Factorization (NNMF) Algorithm Method" was published in 2023. Journal: Appl Bionics Biomech.

In Table 3, the results of Pearson correlation analysis of synergy activation coefficients showed that in the first synergy, the correlation of the synergy activation coefficients between the group with normal vision and the group with blind subjects was 0.431, which shows a moderate similarity (Figure 1(a)). In this synergy in both groups, the peak was in the end stage of walking (swing phase). In blind group, except for the GA muscles, the other muscles were more involved in the synergy, while in the group with normal vision, the anterior tibialis muscle was less involved. In this synergy, the relative weight of external VL muscle in the group with blind subjects increased significantly, as compared to that obtained for the group with normal vision (*P* = 0.023) (Figure 1(b)).

The results also showed that in the second synergy, the correlation of the synergy activation coefficients between two groups was 0.457 (Table 3), showing a moderate similarity between their synergies. In this synergy, the relative weight of BF muscle in the blind group increased significantly compared to that obtained for the normal group (*P* = 0.017) (Figures 1(c) and 1(d)).

Moreover, the results of data analyses indicated that in the third synergy, the correlation of the synergy activation coefficients between two groups was 0.302 (Table 3), reflecting a weak similarity between their synergies. In this synergy, the relative weight of the muscles in the third synergy was not significant for any of the muscles in the groups (Figures 1(e) and 1(f)).

Finally, the results demonstrated that in the fourth synergy, the correlation of synergy activation coefficients between two groups was 0.329 (Table 3), implying a slight similarity between their synergies. In this synergy, the relative weight of VL muscle in the blind group increased significantly (*P* = 0.017) (Figures 1(g) and 1(h)).

## 4. Discussion

The aim of this study was to investigate the effect of vision on muscle synergy in selected lower limb muscles of blind people during walking. The results indicated that there were changes in the muscle synergy model (synergy activation time) and the relative muscle weight of blind people when walking. At the levels of muscle synergy, taking into account the amount of VAF, it was found that, compared with normal-sighted people, the number of muscle synergies in the blind individuals did not significantly change, meaning that the number of muscle synergies in such people remained constant during walking. However, synergy activation time and relative muscle weight in each synergy were different in blind individuals compared to normal-sighted individuals, which was consistent with the findings of previous studies [14].

The article "Measuring the Effect of Vision on the Synergy of Lower Extremity Muscles during Walking using Nonnegative Matrix Factorization (NNMF) Algorithm Method" was published in 2023. Journal: Appl Bionics Biomech.

Yoshida et al. [14] reported the same number of synergies and different relative weights of muscles in each synergy by investigating the effect of impaired vestibular sensory inputs and vision on muscle synergy in sitting-to-standing movement. Yang et al. [25] also expressed similarities in the number of synergies in different sitting-to-standing activities. Desrochers et al. [26] and Takei et al. [27] stated that keeping the number of synergy patterns constant means that the way the CNS controls muscle synergy in healthy and injured individuals is no different.

As the results of the present study showed, despite impaired sensory visual input in the blind individuals, the spinal cord uses similar muscle synergy patterns similar to those in healthy individuals to achieve consistent movements such as walking. Moreover, it was found that the number of synergy patterns in blind individuals was similar to that of healthy individuals, although the patterns of muscle activity in the reported synergies in the two groups were not similar. In other words, the impaired visual input at the CNS level did not change the number of muscle synergies during walking but caused changes in the synergy pattern.

Changes in the pattern of muscle synergy as an effective factor in muscle coordination in the temporal stages of movement can increase the traumatic mechanisms in people with impaired sensory input. By examining muscle synergies obtained for the blind people and people with impaired sensory inputs, a new insight is gained that may change the environmental conditions and the use of new sports tools for these people. Clark et al. [23] examined the synergy of the lower limb muscles in healthy individuals and those with stroke and showed that the number of synergies was the same for both groups and equaled four and that the activation of each synergy in each muscle group would occur at a different stage of the walking cycle. In addition, the relative weight of the muscles was different in the two groups. Saito et al. [28, 29] and Santuz et al. [30] examined the effect of surface slope and walking speed on muscle synergy and showed that the presence of slope and walking speed variables did not change the number of synergies required for walking; however, the trigger points of the synergies and the relative weight of the muscles would change in each synergy. These changes would cause different outputs in the amount of muscle activity. Changes in sensory inputs are generally associated with changes in muscle activation coefficient that modulating the structure of the muscle synergy pattern [30]. Therefore, in this study, it can be argued that differences in the level of sensory feedback in different walking cycles in blind people compared with normal-sighted individuals can be the reason for the change in relative weight and the structure of muscle synergy patterns. As a result, blind people can use other sensory inputs instead of vision to change relative weights in any pattern of muscle synergy during walking [31]. From synergy point of view, with the introduction of different variables, synergy patterns or starting points of any movement pattern in a synergy as well as muscle weight in each synergy can change. By changing the synergy of the muscles, the pattern of muscle activity will also change, and the muscle groups that could be effective in the desired movement are ignored. Therefore, with proper weighting in that synergy, movements can be maintained and controlled. However, in most studies on muscle synergy, walking at different speeds, walking at different levels, walking with different disorders such as stroke, Parkinson's disease, senility, etc., eight or even more muscles have been studied at the same time. However, based on the VAF value, four muscle synergies were extracted for walking in different conditions [11, 23]. They have concluded that increasing the number of muscles can lead to the extraction of a more accurate number of muscle synergies. However, in the present study, while only five lower-limb muscles were examined, four muscle synergies with different activity patterns and different relative muscular weights were observed in the both blind and normal-sighted groups during walking.

The article "Measuring the Effect of Vision on the Synergy of Lower Extremity Muscles during Walking using Nonnegative Matrix Factorization (NNMF) Algorithm Method" was published in 2023. Journal: Appl Bionics Biomech.

### 4.1. Limitations and Future Work

This paper conducted a preliminary study on the muscle synergy of lower extremity muscles between the two groups during walking. Despite some interesting achievements, there are still some limitations that need to be addressed in future work.

First, only nine healthy adult male subjects and nine adult male blind were involved in this study. The small number of subjects, for example, may limit the statistical results. Thus, more subjects should be recruited for future work. Second, the datasets we used included only five muscles, which may limit our understanding of neuromuscular control strategies, especially in complex motions such as walking. More muscles should be considered for the future.

## 5. Conclusion

Based on the findings of the present study, it can be concluded that the lack of visual input in blind people compared to people with normal vision during walking does not have a significant effect on the structure and number of muscle synergies; however, the relative weight of muscles in each synergy can change. It seems that adaptations in the strategy of the nervous system to recruit and activate the muscles affect the pattern of walking and the use of other sensory systems, which increases motor performance in the blind people and avoids injuries in the vision loss conditions. In future studies, we suggest investigating the lower limb muscles synergy in healthy people with eyes open, eyes closed, and blind people.

## Figures and Tables

**Figure 1:** (a, c, e, and g) Mean components of synergy activation coefficients from the breakdown of EMG signals into four synergies in the groups with normal vision and blind subjects; (b, d, f, and h) mean values of muscle synergy with standard deviation in the two groups with normal vision and blind subjects ( ^*∗*^ shows a significant difference in *P* < 0.05).

**Table 1:** Mean and standard deviation of subjects' demographic variables in the studied groups.

	Groups		Sig.
	Blind	Normal vision	
Age (years)	24.70 ± 5.5	23.90 ± 4.9	0.72
Height (m)	1.71 ± 0.05	1.75 ± 0.04	0.06
Weight (kg)	68.10 ± 10.7	78.50 ± 7.53	0.09
BMI (kg/m^2^)	23.33 ± 3.8	25.46 ± 2.28	0.15

Abbreviation: BMI: body mass index (weight/height^2^).

**Table 2:** VAF of control group and blind group for different number of synergy.

Number of synergy	Normal group	Blind group
1	0.591 ± 0.1	0.610 ± 0.073
2	0.746 ± 0.74	0.737 ± 0.73
3	0.836 ± 0.83	0.806 ± 0.8
4	0.950 ± 0.85	0.923 ± 0.86

**Table 3:** Results from Pearson correlation analysis of synergy activation coefficients.

Blind				
Normal	Synergy 1	Synergy 2	Synergy 3	Synergy 4
Synergy 1	**0.431**	0.548	0.005	0.044
Synergy 2	0.430	**0.457**	0.346	0.032
Synergy 3	0.465	0.567	**0.302**	0.264
Synergy 4	0.619	0.618	0.166	**0.329**

Bold values signify the correlation between two groups.

## Data Availability

The EMG data used to support the findings of this study are available from the corresponding author upon request.

## References

[1] Chvatal S. A., Ting L. H. (2013). Common muscle synergies for balance and walking. *Frontiers in Computational Neuroscience*.

[2] d’Avella A., Bizzi E. (2005). Shared and specific muscle synergies in natural motor behaviors. *Proceedings of the National Academy of Sciences*.

[3] Ting L. H., Chvatal S. A., Danion F., Latash M. (2010). Decomposing muscle activity in motor tasks methods and interpretation. *Motor Control: Theories, Experiments, and Applications*.

[4] Tresch M. C., Jarc A. (2009). The case for and against muscle synergies. *Current Opinion in Neurobiology*.

The article "Measuring the Effect of Vision on the Synergy of Lower Extremity Muscles during Walking using Nonnegative Matrix Factorization (NNMF) Algorithm Method" was published in 2023. Journal: Appl Bionics Biomech.

[5] Barimani S., Maleki A., Fallah A. (2014). Influence of mechanical terms in quantifying muscle synergy during cycling for FES rehabilitation applications. *Iranian Journal of Biomedical Engineering*.

[6] Bernshteĭn N. A. (1967). *The Co-Ordination and Regulation of Movements*.

[7] Lacquaniti F., Ivanenko Y. P., Zago M. (2012). Development of human locomotion. *Current Opinion in Neurobiology*.

[8] Eslamy M., Alipour K. (2019). Synergy-based Gaussian process estimation of ankle angle and torque: conceptualization for high level controlling of active robotic foot prostheses/orthoses. *Journal of Biomechanical Engineering*.

[9] Nakamura T. (1997). Quantitative analysis of gait in the visually impaired. *Disability and Rehabilitation*.

[10] Timmis M. A., Scarfe A. C., Tabrett D. R., Pardhan S. (2014). Kinematic analysis of step ascent among patients with central visual field loss. *Gait & Posture*.

[11] Nougier V., Bard C., Fleury M., Teasdale N. (1997). Contribution of central and peripheral vision to the regulation of stance. *Gait & Posture*.

[12] Cappellini G., Ivanenko Y. P., Poppele R. E., Lacquaniti F. (2006). Motor patterns in human walking and running. *Journal of Neurophysiology*.

[13] Hagio S., Fukuda M., Kouzaki M. (2015). Identification of muscle synergies associated with gait transition in humans. *Frontiers in Human Neuroscience*.

[14] Yoshida K., An Q., Yozu A. (2018). Visual and vestibular inputs affect muscle synergies responsible for body extension and stabilization in sit-to-stand motion. *Frontiers in Neuroscience*.

[15] Huang Y., Song R., Chen W. The effects of different tracking tasks on muscle synergy through visual feedback.

[16] Ivanenko Y. P., Poppele R. E., Lacquaniti F. (2004). Five basic muscle activation patterns account for muscle activity during human locomotion. *The Journal of Physiology*.

[17] Martino G., Ivanenko Y. P., d’Avella A. (2015). Neuromuscular adjustments of gait associated with unstable conditions. *Journal of Neurophysiology*.

[18] Hermens H. J., Commission des Communautés Européennes (1999). *SENIAM: European Recommendations for Surface Electromyography: Results of the SENIAM Project*.

[19] Steele K. M., Tresch M. C., Perreault E. J. (2013). The number and choice of muscles impact the results of muscle synergy analyses. *Frontiers in Computational Neuroscience*.

[20] Chen J.-J. J., Shiavi R. G., Zhang L.-Q. (1992). A quantitative and qualitative description of electromyographic linear envelopes for synergy analysis. *IEEE Transactions on Biomedical Engineering*.

[21] Hallemans A., Ortibus E., Meire F., Aerts P. (2010). Low vision affects dynamic stability of gait. *Gait & Posture*.

The article "Measuring the Effect of Vision on the Synergy of Lower Extremity Muscles during Walking using Nonnegative Matrix Factorization (NNMF) Algorithm Method" was published in 2023. Journal: Appl Bionics Biomech.

[22] Lee D., Seung H. S., Leen T., Dietterich T., Tresp V. (2000). Algorithms for non-negative matrix factorization. *Advances in Neural Information Processing Systems*.

[23] Clark D. J., Ting L. H., Zajac F. E., Neptune R. R., Kautz S. A. (2010). Merging of healthy motor modules predicts reduced locomotor performance and muscle coordination complexity post-stroke. *Journal of Neurophysiology*.

[24] Mukaka M. M. (2012). A guide to appropriate use of correlation coefficient in medical research. *Malawi Medical Journal*.

[25] Yang N., An Q., Yamakawa H., Tamura Y., Yamashita A., Asama H. (2017). Muscle synergy structure using different strategies in human standing-up motion. *Advanced Robotics*.

[26] Desrochers E., Harnie J., Doelman A., Hurteau M.-F., Frigon A. (2019). Spinal control of muscle synergies for adult mammalian locomotion. *The Journal of Physiology*.

[27] Takei T., Confais J., Tomatsu S., Oya T., Seki K. (2017). Neural basis for hand muscle synergies in the primate spinal cord. *Proceedings of the National Academy of Sciences*.

[28] Saito A., Tomita A., Ando R., Watanabe K., Akima H. (2018). Muscle synergies are consistent across level and uphill treadmill running. *Scientific Reports*.

[29] Saito A., Tomita A., Ando R., Watanabe K., Akima H. (2018). Similarity of muscle synergies extracted from the lower limb including the deep muscles between level and uphill treadmill walking. *Gait & Posture*.

[30] Santuz A., Ekizos A., Eckardt N., Kibele A., Arampatzis A. (2018). Challenging human locomotion: stability and modular organisation in unsteady conditions. *Scientific Reports*.

[31] Maurer C., Mergner T., Bolha B., Hlavacka F. (2000). Vestibular, visual, and somatosensory contributions to human control of upright stance. *Neuroscience Letters*.

